The article "Application of Dynamic Enhanced Magnetic Resonance Imaging in the Diagnosis of Hematological Malignancies" was retracted in 2023. Reasons: signs of a paper mill; suspected computer-generated content; unreliable results or conclusions; lack of ethics approval or compliance.

# Application of Dynamic Enhanced Magnetic Resonance Imaging in the Diagnosis of Hematological Malignancies

**DOI:** 10.1155/2021/4623850

**Published:** 2021-12-23

**Authors:** Yanping Shao, Xueping Bao, Caifang Song, Danping Cui

**Affiliations:** ^1^Department of Hematology, Taizhou Hospital of Zhejiang Province Affiliated to Wenzhou Medical University, Taizhou, Zhejiang 317000, China; ^2^Taizhou Hospital of Zhejiang Province Affiliated to Wenzhou Medical University, Taizhou, Zhejiang 317000, China; ^3^Department of Gastroenterology, Taizhou Hospital of Zhejiang Province Affiliated to Wenzhou Medical University, Taizhou, Zhejiang 317000, China; ^4^Department of Geriatrics, Taizhou Hospital of Zhejiang Province Affiliated to Wenzhou Medical University, Taizhou, Zhejiang 317000, China

## Abstract

The use of dynamic enhanced magnetic resonance imaging technology can effectively explore the diagnosis and clinical application of hematological malignancies. This paper selected 60 patients with hematological malignancies from 2015 to 2019; all of whom were diagnosed with hematological malignancies, including 40 men and 20 women, aged between 40 and 77 years. The main clinical manifestations of the patient are hematological malignancies, fever, and other symptoms. We used Siemens 3.0T to perform MRI and dynamic enhanced MRI examinations on 30 patients with hematological tumors. The PACS system was used to collect and organize clinical data. All patients were pathologically confirmed and clinically diagnosed with hematological malignancies. Based on the clinical data of the patients, retrospective analysis and summary were conducted and the clinical manifestations of hematological malignancies were discussed. The results showed that the diagnostic accuracy of 30 cases of dynamic enhanced MRI was 100%, while the diagnostic accuracy of ordinary MRI was lower than that of dynamic enhanced MRI, *P* < 0.05, and the difference was statistically significant. In addition, compared with dynamic enhanced MRI and MRI, *P* > 0.05, the difference was not statistically significant. Therefore, the application of dynamic enhanced MRI in the diagnosis of hematological malignancies is valuable.

## 1. Introduction

With the development of urbanization, industrialization, and the advent of population aging, the incidence rate is on the rise. Malignant tumors have brought serious harm to human health. Researching malignant tumors to design more effective treatment plans is an important direction of modern medicine development. With the invention and application of new technologies, the overall diagnosis level has significantly improved, and with the clinical application of new drugs, the treatment level has improved significantly [1]. The scientific and effective application of various diagnostic indicators to make them play the best guiding role in the treatment is a challenge facing the field of hematological malignancies. Diagnosis is the prerequisite for achieving accurate treatment. Only accurate diagnosis can play its clinical guiding role, and the implementation of magnetic resonance imaging is the basis for accurate diagnosis [2]. The prospect of new technology is very bright, but the current application is not very satisfactory.

Dynamic enhanced magnetic resonance imaging (DE-MRI) is a functional imaging method that noninvasively evaluates the characteristics of tissues and tumor blood vessels through intravenous injection of contrast medium. The current MRI-enhanced contrast agents include small molecule contrast agents that can quickly diffuse into the extracellular space (relative molecular mass <1000). The small molecule contrast agent DCE-MRI technology has successfully entered the clinical application stage and has played an important role. The DCE-MRI technology is in the early stage of clinical trials and clinical applications. In the process of research on malignant tumors by researchers and doctors, dynamic contrast-enhanced magnetic resonance imaging as an imaging technique that reflects the characteristics of tissue hemodynamics has received more and more clinical applications [3, 4]. In DE-MRI imaging, a paramagnetic substance has usually been injected into the patient's body through an intravenous injection, which results in a shortened T1 time during tissue imaging. Repeated imaging is used to track the diffusion of the contrast agent into the tissue over time. This can reflect hemodynamic information such as microangiogenesis and permeability of living tumors and plays an important role in the diagnosis and research of malignant tumors. The DE-MRI image analysis is mainly carried out in two aspects: (1) analysis pixel by pixel in the spatial domain and (2) time domain analysis in the image sequence, by analyzing the changes in the concentration of the local spatial contrast agent, calculating the relevant hemodynamic parameters.

Today, the level of informatization is getting higher, and the massive growth in medical imaging data makes it more necessary to use computers for automatic processing or to extract key information for doctors, thereby promoting the development of computer-aided diagnosis. Dynamically enhanced MRI uses imaging, medical image processing technology, and other possible physiological and biochemical methods, which improves the accuracy of lesion location [5]. The use of dynamic enhancement of MRI can speed up the diagnosis process, reduce the rate of misdiagnosis, improve the quantitative evaluation results, and help correct the doctor's subjective diagnosis error [6]. Nevertheless, the application of dynamic enhancement MRI technology in the field of DE-MRI imaging is only relatively mature in multiple myeloma research, and the clinical application of other diseases needs further development [7]. Therefore, how to improve and strengthen the MRI technology so that the DE-MRI image processing and analysis field has better clinical promotion is the key to promoting the development of related technologies.

We transfer all the collected original images to the Extended MR Workspace (EWS) workstation provided by Philips, which contains the Functool toolkit for postprocessing all images. The film was read by two experienced MRI diagnostic doctors, and the pathological results were not known before the film. When there is a disagreement, it will be decided by the two doctors after mutual consultation. If the lesion is multiple, the largest lesion diameter is included when analyzing the MRI image. The data was sorted and summarized, a database was established with Excel 2010, SPSS 24.0 was used for statistical analysis of all the data, the measurement data was tested for normal distribution by the Kolmogorov–Smirnov method, and the homogeneity of variance test was performed by the Leneve method. If the data conform to the normal distribution and the variance is homogeneous, then the paired-sample *t*-test or the two-independent-sample *t*-test will be used. If the data does not conform to the normal distribution and the homogeneity of variance, the nonparametric rank-sum test is used. The comparison of count data, morphology, and TIC curve type was analyzed by *X*^2^ test and Fisher exact probability method. *P* < 0.05 is considered the difference to be statistically significant; *P* > 0.05 is considered the difference not to be statistically significant. We draw receiver operating characteristic curves for statistically significant indicators. Specifically, the technical contributions of this paper can be summarized as follows:

  First, this paper innovatively uses dynamic enhanced magnetic resonance imaging technology to explore the diagnosis and clinical application of hematological malignancies.
  Second, through Siemens 3.0T, we performed MRI and dynamic enhanced MRI on 30 patients with hematological tumors and used the PACS system to collect and organize clinical data.
  Third, this paper conducts a retrospective analysis and summary to discuss the clinical manifestations of hematological malignancies. The results prove that the application of dynamic enhanced MRI in the diagnosis of hematological malignancies is very effective.

## 2. Materials and Methods

### 2.1. General Information

Sixty patients with hematological malignancies who came to our hospital from January 2015 to December 2019 were selected as the research subjects. All of them had fever, bone pain, weight loss, and symptoms such as low fever; all were diagnosed as hematological malignancies. Patients who had low compliance and had mental disorders were excluded. According to the order of visits, they were divided into the control group and experimental group, each with 30 cases. In the control group, there were 20 males and 10 females; they were 46–68 years old, with an average of 48.5 ± 1.5 years old. In the experimental group, there were 20 males and 10 females. They were 46–68 years old, with an average of 48.7 ± 1.4 years old. There was no statistically significant difference between the two groups of patients in terms of condition, age, and other pieces of information (*P* > 0.05), and they were comparable.

### 2.2. Method

Patients in the control group were given MRI examinations. First, the vertebral bodies of the patients were scanned, and the thickness was controlled at 5 mm. Secondly, the imaging staff carefully observe the soft tissue window and bone window of the patient's image. Finally, a small number of patients with hematological malignancies were given meglumine by intravenous injection, then enhanced scanning was performed, and images were acquired to diagnose their condition [8]. The experimental group was diagnosed with MR, and the patients were scanned with Siemens 3.0T MR instrument, combined with the patient's condition, including T2W1, axial FSE, and SE sequence T1W1. All subjects underwent a full spine scan and moved the bed according to the needs of the scan. The relevant parameters of the scan include the following: the sagittal scan layer thickness is 3 to 4 mm, and the separation distance is 0.35 mm. Then, 10∼12 ml of diethylenepentamine gadolinium acetate is used to give the patient, and then the enhanced scan is performed, *b* = 700 mm/s, and the number of excitations is 2 to 3 times [9].

### 2.3. Statistical Methods

The software SPSS 19.8 was used to process the data, the measurement data was expressed as *x* ± *s*, and the *t*-test was used; the count data was expressed in 97%, and the *χ*^2^ test was used; *P* < 0.05 indicates that the difference is statistically significant.

## 3. Modeling and Simulation Results

### 3.1. DE-MRI

#### 3.1.1. MRI

DE-MRI uses a fast T1WI sequence to scan the lesions in multiple phases and measures the changes of T1 signal intensity before and after intravenous bolus injection of contrast medium, which obtains tissue perfusion, capillary surface area, vascular permeability, and dynamic enhancement curves through postprocessing techniques in Figure 1. Such as a series of semiquantitative and quantitative parameters can more objectively reflect the pathophysiological characteristics of the disease. T1WI sequence usually uses gradient-echo sequence and saturation recovery/reversal recovery rapid imaging sequence, such as rapid three-dimensional volumetric interpolated breath-hold examination (VIBE), multiple myeloma, and liver acquisition with volume acceleration (LAVA) sequence, and tries to avoid the influence of T2 and T2∗ signals.

The basic principle of magnetic resonance imaging is to place the object under inspection in a strong magnetic field, and the magnetic moments of certain protons are arranged along the magnetic field and move around the direction of the magnetic field at a certain frequency [10]. On this basis, a radio frequency pulse with the same frequency as the motion of the proton is used to excite the proton magnetic moment to cause energy level conversion, release energy, and generate a signal during the relaxation of the proton. The receiving coil of MRI acquires the above-mentioned signals, then amplifies them through an amplifier, and inputs them to a computer for image reconstruction, thereby obtaining the magnetic resonance images we need. In addition to the charge and mass of the nucleus, about half of the nuclei of the elements can spin. Since the nucleus is a positively charged particle, its spin will generate a small magnetic field. The total magnetic moment ${\overset{⟶}{\mu }}_{j}$ and the total angular momentum ${\overset{⟶}{P}}_{k}$ have the following relationship:

(1) $$\begin{array}{c} {\overset{⟶}{\mu }}_{k}=-g\frac{E}{2m_{e}}{\overset{⟶}{P}}_{k}=g\frac{2\pi \mu_{B}}{h}{\overset{⟶}{P}}_{k}=\gamma {\overset{⟶}{P}}_{k}, \end{array}$$

where *E* is the Delang factor, *e* and *m*_*e*_ are the electronic charge and mass, *μ*_*B*_ is called the Bohr magneton, and *R* represents the gyromagnetic ratio of the atom. For nuclei with nonzero spin, the nuclear magnetic moment ${\overset{⟶}{\mu }}_{j}$ and spin angular momentum ${\overset{⟶}{P}}_{k}$ also have the following relationship:

(2) $$\begin{array}{c} {\overset{⟶}{\mu }}_{I}=-g_{N}\frac{E}{2m_{p}}{\overset{⟶}{P}}_{k}=g_{N}\frac{2\pi \mu_{N}}{h}{\overset{⟶}{P}}_{k}=\gamma {\overset{⟶}{P}}_{k}. \end{array}$$

According to quantum theory, there is a quantum mechanical system of nuclear spin and nuclear magnetic moment. In an external magnetic field *B*_0_, the energy level will undergo Zeeman splitting. There is an energy difference Δ*E* among adjacent energy levels. When external conditions provide the same magnetic energy Δ*E*, it will cause a phase. The magnetic dipole transition between adjacent Zeeman energy levels, for example, the energy difference Δ*E*=(*RD*_0_*h*/2*π*) of the Zeeman energy level, is that the hydrogen nucleus emits a photon of energy *hν*. At that time, the hydrogen nucleus will absorb this photon and transition from a low Zeeman energy level to a high Zeeman energy level [11]. It can be seen from Figure 1 that nuclear magnetic resonance occurs and the condition is that the circular frequency of electromagnetic waves is as follows:

(3) $$\begin{array}{c} \omega_{0}=RD_{0}. \end{array}$$

When nuclei with spins are in a uniform fixed magnetic field, they will interact. As a result, the spin axis of the nuclei will move along the circular orbit in the magnetic field. This movement is called precession. The precession frequency *ω*_0_ of the spin nucleus is proportional to the applied magnetic field strength *H*_0_, where *R* is the gyromagnetic ratio, which is a constant characterized by different nuclei; that is, different nuclei have their own inherent gyromagnetic ratio *γ*, which is the basis for qualitative analysis using nuclear magnetic resonance spectrometer. It can be seen from the above formula that if the spin nucleus is in a fixed magnetic field with a magnetic field strength of *H*_0_ and tries to measure its precession frequency *ω*_0_, the gyromagnetic ratio *γ* can be obtained, thereby achieving the purpose of qualitative analysis. At the same time, you can keep *ω*_0_ unchanged, measure *H*_0_, find *γ*, and realize qualitative analysis.

In recent years, with the development of magnetic resonance imaging equipment software and hardware, especially the development of gradient magnetic field technology, MR scanning speed is getting faster and faster. A new dynamic enhancement MRI method—contrast-enhanced dynamic enhancement MRI (DE-MRI)—came into being [12]. Dynamic enhanced MRI has a wide range of applications and strong practicability, especially for the chest blood vessels (including heart and large blood vessels and pulmonary blood vessels), abdominal blood vessels, and pulsating limb blood vessels in the physiological movement area. For example, in limb vascular imaging, dynamic enhanced MRI can overcome the shortcomings of ordinary TOF and PCA techniques such as long imaging time, overevaluation of vascular stenosis, and obvious pulsation artifacts, which has high spatial resolution.

#### 3.1.2. Structure and Composition of the 400 MHz MRI Spectrometer

Figure 2 shows the structure and composition of 400 MHz MRI spectrometer. The whole system is composed of the machine body, main cabinet, and console. The electromagnetic signal from the console is converted into an analog signal by the main cabinet to control the process of the body to complete the experiment. The analog signal collected by the body detector is converted into an electrical signal by the main cabinet, and the range is to the console and saved as a nuclear magnetic spectrogram. The body is composed of a superconducting magnet, sampler, detector, and so on [13]. The superconducting magnet is the core component of a nuclear magnetic spectrometer, which is used to generate the magnetic field required for the operation of the instrument. There are 72 sets of coils around the superconducting magnet. The superconducting magnet is surrounded by a cooling pool of liquid nitrogen and liquid helium to maintain the low-temperature environment required by the superconducting magnet. The instrument is equipped with a 60-position autosampler, which can arrange sequential experiments. The detector consists of a transmitter coil and a receiver coil to detect the nuclear magnetic signal of the sample.

Dynamic enhanced MRI uses a fast gradient-echo sequence of very short TR and very short TE. In the case of such short TR and TE, the longitudinal magnetization of various tissues is very small, and the signal strength is also very small. If a paramagnetic contrast agent is injected into the blood vessel, the T1 relaxation time of the blood will be extremely shortened. The T1 relaxation time of the blood vessel is much shorter than the T1 relaxation time of the background tissue. The blood has a high signal, forming a strong contrast between the blood vessel and the background [14].

In dynamic enhanced MRI, digital subtraction technology can also be used to subtract the corresponding pixel signal intensity between the two sets of images obtained before and during the injection of gadolinium contrast agent. Subtractive dynamic enhanced MRI is compared with nonsubtractive dynamic enhanced MRI which improves the contrast/noise ratio and improves the display of blood vessels.  Figure 3 shows the signal recognition of DE-MRI. The advantages of magnetic resonance imaging are nonradiation and noninvasive and multidirectional and arbitrary-angle imaging. Many imaging parameters have strong diagnostic significance for the location and nature of the lesion; the high resolution of soft tissues is increasingly receiving clinical attention and welcome.

Due to the increase in scanning speed, patients can perform multiple volume acquisitions of organs of interest in one breath-hold, which improves the time resolution of lesion detection. Alternatively, high scanning speed can be exchanged for high-resolution scanning to improve spatial resolution.

### 3.2. Clinical Trials and Results Analysis

Research progress of dynamic enhancement MRI is based on DE-MRI images of malignant tumors. The application of dynamic enhancement MRI in the field of DE-MRI imaging can mainly include the following steps: ① image preprocessing; ② segmentation of interesting areas; ③ feature extraction; ④ classification and tumor region recognition. As shown in Figure 4, the process of the entire dynamic enhancement MRI system is shown.

#### 3.2.1. Image Preprocessing

Image preprocessing mainly includes noise reduction and image sequence registration. Its main purposes are as follows: (1) DE-MRI imaging time is short, and the image signal-to-noise ratio is low, so the image noise reduction is extra important. (2) The patient is undergoing DCE. The movement of the body due to breathing or other reasons during the MRI imaging process will cause coordinate deviations between DE-MRI images, which must be corrected. Most researchers mainly use a Gaussian low-pass filter to reduce noise [14], but the Gaussian low-pass filter will smooth the image, causing the resolution of the image to decrease, so a more ideal filtering method is required. As shown in Figure 4, a summary of several commonly used image noise reduction is given, and the advantages and disadvantages of each algorithm are briefly summarized. For the research on motion compensation of DE-MRI image sequence, the classification of commonly used image registration methods is given, and the advantages and disadvantages of each method are summarized.

Image preprocessing can reduce image noise, correct errors generated in the imaging process, improve image quality, and provide more accurate information. It can be seen from Table 1 that the main problem of the existing methods is that the noise reduction process may reduce the spatial resolution of the image and cause the loss of image information. Therefore, future research should focus on how to minimize the loss of image information while ensuring the noise reduction effect, and it can be seen that, in the existing registration algorithms, the registration accuracy is affected by various factors. In the future, when studying the new DE-MRI image sequence registration, it is necessary to distinguish whether the algorithm used is actually suitable for rigid body registration or nonrigid body registration, and at the same time, the factors that affect the registration accuracy should be identified.

#### 3.2.2. Tumor Area Division

After denoising the image and correcting the motion error of the image sequence, preliminary segmentation of the tumor region is needed to reduce the computational cost. The main methods are manual segmentation and automatic segmentation. The manual division has performed by a doctor, so the accuracy is limited by the doctor's clinical experience, which is time-consuming. In recent years, the application of dynamic enhanced MRI for automatic segmentation has gradually attracted people's attention. Among them, the more common methods are clustering and the hybrid algorithm that combines the aforementioned methods. As shown in Figure 5, the advantages and disadvantages of these algorithms are summarized.

Tumor area segmentation can increase the speed of image processing and eliminate unnecessary backgrounds. Currently, the commonly used tumor region segmentation for DE-MRI images is shown in Table 2. Among them, the clustering method is well-researched and the process is simple, but the results of the image segmentation obtained are often not ideal. Compared with the traditional clustering algorithm, the image segmentation accuracy of the horizontal set, Markov random field, artificial neural network, and other algorithms has been significantly improved, but due to the higher number of algorithm iterations, the calculation time has also increased significantly [15]. Therefore, in the future, when selecting the tumor region segmentation for DE-MRI images, it is necessary to weigh the pros and cons of each method and find the optimal algorithm with shorter time-consuming and higher segmentation accuracy.

#### 3.2.3. Feature Extraction

In order to analyze the tumor area, such as judging whether the area is a diseased area, it is often necessary to estimate certain features or characteristics of the ROI area, which is also the extraction of the characteristics of the tumor area. Dynamically enhanced MRI uses a computer to replace or assist the human brain to identify tumor areas, and the ability of features to express data determines the ultimate effect that dynamic enhanced MRI can achieve to a certain extent [16]. Features with strong expression ability should well characterize the differences between different tissues (tumor area and nontumor area), and at the same time, the dimension should not be too high, to ensure the efficiency of calculation. The common features of DE-MRI images mainly include morphological characteristics, texture characteristics, hemodynamic curve characteristics, and pharmacokinetic characteristics. As shown in Table 2, the related literature is given, and the advantages and disadvantages of these features are briefly summarized.

As shown in Table 2, among the common features of DE-MRI images listed, morphological features and texture features are commonly used in image processing, while hemodynamic and pharmacokinetic features are DE-MRI images' unique characteristics [17]. Compared with morphological and texture characteristics, hemodynamic characteristics and pharmacokinetic characteristics can reflect the change characteristics of the DE-MRI image sequence. Therefore, the classifier trained as a feature has a better classification and recognition effect. It should be pointed out that the features listed in Table 2 are only part of the feature information contained in DE-MRI images. Therefore, the focus of future research is to find more and better features to characterize the characteristics of DE-MRI images.

### 3.3. Results

#### 3.3.1. Flat Sweep

Of the 30 patients, 20 had a single lesion and 10 had multiple lesions. A total of 67 lesions were found, of which 54 were located in the right lobe of the liver and 13 were located in the left lobe of the liver.

19 lesions were round and 48 were round or irregular. The size of the lesion is 7∼85 mm, average 25–11 mm; 15 lesions > 30 mm. Seven cases were complicated by liver cysts.

Dynamic enhanced scanning adopts 3D-FLASH plus fat suppression sequence TR/TE = 4.42/1.46 ms in Table 3; FOV = 320 mm. The matrix is 320 × 512. Layer thickness is 0.8 mm, and interval is 0.18 mm. The inversion angle is 12°. The scanning range includes the whole cavity which is repeatedly scanned 6–8 times continuously, with an interval of 20 seconds after the first scan, for the injection of contrast agent, and the scanning time is 7–9 minutes as in Table 3.

#### 3.3.2. Dynamic Enhancement

In 30 patients, 46 lesions showed discontinuous marginal nodular enhancement, which filled the center of the lesion with time, and 21 lesions showed irregular or rapid peripheral enhancement. Early dynamic enhancement of 3 lesions (equivalent to arterial phase) showed the blood supply artery, 5 lesions showed early visualization and drainage vein (Figure 6), and 14 tumors around the enhancement (4 showed irregular edge enhancement, and 10 showed liver pack wedge strengthening under the membrane) [18]. During the dynamic scanning period, 27 lesions were completely filled and enhanced (Figure 6(d)), and 40 lesions were not completely filled and enhanced.

#### 3.3.3. Delayed Enhanced Scanning

The delay time is 6–9 min, average (7.3 ± 0.8) min. 53 lesions were completely filled and enhanced, of which 37 lesions were relatively high signals, and 16 lesions had equal signals. The filling area of 14 lesions showed high signal or isointensity, and the unfilled area showed patchy or crack-like low signal (Figure 7).

After the examination of 30 multiple myeloma patients, the results of the dynamic time-signal intensity curve were 3 cases with type I curve, 17 cases with type II curve, and 20 cases with type III curve. See Table 1 for details. Hematological malignancies can occur at any age, and most of them occur in adults, most commonly between 46 and 68 years old. There are more males than females. The multiple myeloma varies in size, and those over 40mm are rare.

#### 3.3.4. Comparison of Results

Pathologically, the cut surface of multiple myeloma is filled with blood. The microscopic examination of of Multiple Myeloma shows that it is composed of cystic blood sinusoids or blood pools of varying sizes. There is a fibrous tissue septum between the blood sinusoids. The blood flows slowly in it, mostly from the edge of the tumor to the center [19]. The nodules around the lesion are enhanced at an early stage and filled to the center of the lesion despite the prolonged time. The rapid filling after enhancement seems to relate to the size of multiple myeloma. The proportion of multiple myeloma is about 16%, but it accounts for 42% of the enhancement mode of small hemangioma. During the dynamic enhancement period, 41% (25/60) of multiple myeloma were seen to be fully filled and enhanced. Compared with the surrounding normal multiple myeloma, it was a high signal or iso-signal. 19% (11/60) of the lesions showed low signal shadow with an incomplete filling of flaky or fissure-like enhancement, which may be related to liquefaction, hemorrhage, thrombosis, and extensive hyaline degeneration and fibrosis in the multiple myeloma in Figure 8. Hepatic hemangioma has often accompanied by an arteriovenous short circuit, which was to be seen in malignant liver tumors in the past. Figure 8 shows the comparing results of MRI and DE-MRI.

In the early stage of dynamic enhanced MRI scan, 25% (15/60 lesions) of multiple myeloma showed temporary substantial enhancement. 67% (40/60) of which were related to the existence of increased erythrocyte sedimentation rate [20]. Dynamic enhanced MRI in the early stage of MRI found that 50.1% (31/60 lesions) of multiple myeloma showed temporary substantial enhancement in the adjacent area, and it was more common in rapidly enhancing lesions [3]. In this group, 8% (5/60) of the lesions showed enhancement of early venous visualization, and 23% (14/60) multiple myeloma parenchyma enhanced. Dynamic enhanced MRI scan found that 49% (28/60) of multiple myeloma showed temporary enhancement around the tumor, which has mainly manifested as enhanced early subcapsular wedge enhancement and increased erythrocyte sedimentation rate. This change is more seen in small lesions that rapidly strengthen. It is inferred that small multiple myelomas with rapid strengthening are usually in a hyperhemodynamic state, which contains large and rapid drainage that causes the tumor to rapidly strengthen the larger arterial blood flow and causes early increased erythrocyte sedimentation rate and enhancement of the surrounding parenchyma.  Figure 9 shows the different segments of multiple myeloma MRI.

In most cases, it is not difficult to make a differential diagnosis of multiple myeloma on imaging examination. The T2WI imaging of the MRI of a typical multiple myeloma is characteristic. With the extension of TE, the signal increases, with a typical/bulb sign 0. The enhancement is manifested as uniform enhancement in the arterial phase or enhancement of the marginal nodules, which is consistent with the enhancement of adjacent arteries, which is delayed. At the time, the enhancement of the lesion is obvious, while for liver cancer, it is the enhancement performance of/fast forward and fast out 0. Neuroendocrine tumors and metastases of breast and colon cancers show strong T2 signals [5]. Delayed enhancement of MRI in some malignant tumors with rich blood supply is similar to a few atypical multiple myeloma. Once the hepatic hemangioma shows that the enhanced area will not disappear, the combined consideration of multiple imaging signs will help the differential diagnosis. Multiple Myeloma is manifested as increased erythrocyte sedimentation rate and wedge-shaped or irregular enhancement around the tumor, which is more common in small rapidly enhancing multiple myeloma and unevenly enhancing lesions. The appearance of this sign is conducive to the differential diagnosis of multiple myeloma.

### 3.4. Discussion

DE-MRI has evolved from simple qualitative analysis to multiparameter quantitative analysis, and clinical research has expanded from the nervous system to the whole body. Among the most widely used tumor imaging, the research of DE-MRI covers various aspects such as the differential diagnosis of benign and malignant lesions, clear tumor grading, evaluation of efficacy and prognosis, and detection of tumor recurrence. In recent years, clinical research on tumor antivascular therapy has been widely carried out. Traditional biomarker technology is difficult to evaluate the efficacy of antitumor vascular drugs early. The application of quantitative parameters related to DE-MRI which can help in terms of tumor morphology, vascular function, and cell metabolism dynamic observation of the treatment effect is convenient for timely adjustment of drug dosage and optimization of the treatment plan.

#### 3.4.1. Tumor Diagnosis and Differential Diagnosis

DE-MRI is widely used in the differential diagnosis of benign and malignant tumors in various systems. Among them, the diagnosis of multiple myeloma, prostate cancer, glioma, and other solid tumors has been a research hotspot in recent years in Figure 10. The microenvironment such as hypoxia and weak acidity in malignant tumors and the activation of oncogenes can induce the expression of vascular endothelial growth factor (vascular endothelial growth, VEGF) and other vascular endothelial genes to increase, thereby stimulating the massive formation of abnormal blood vessels in the tumor. New tumors have tortuous and irregular microvessels, incomplete basement membranes, and widened endothelial cell gaps, leading to increased tumor vascular resistance and microvascular permeability. Therefore, the quantitative parameter values reflecting tumor area tissue perfusion and vascular endothelial cell integrity have abnormal changes. A series of studies have shown that there are significant differences in the Ktrans value, initial enhancement time, maximum enhancement level, and enhancement curve of prostate cancer and prostate hyperplasia tissue. In recent years, there have been many studies on gliomas. The results showed that Vp (plasma volume fraction) is the quantitative parameter with the highest sensitivity and specificity in the differential diagnosis of the two. The accuracy of the differential diagnosis between the two when the Ktrans value and the Vp value are combined can reach 96%.

#### 3.4.2. Tumor Pathological Type and Grade

Tumor tissues differentiated from different tissues have different biological characteristics. Because the pharmacokinetics of contrast agents in different pathological tissues is different, DE-MRI can reflect the essential differences of different pathological types of tumors. DCEMRI quantitative analysis method is to retrospectively study squamous cell carcinoma, undifferentiated carcinoma, and lymphoma that occurred in the head and neck, and the results showed that the Ktrans value of undifferentiated carcinoma was significantly higher than that of the other two malignancies. Tumors and the Ktrans values of the three tumors are consistent with VEGF expression levels. The higher the grade and the poorer the level of differentiation of the same pathological type of tumor, the higher the permeability of the blood vessel wall and the ratio of extracellular extravascular space and the faster the contrast medium exchange rate (Ktrans).

#### 3.4.3. Efficacy Evaluation and Prognosis Judgment

Radiotherapy and chemotherapy are indispensable links in tumor treatment, but the therapeutic effect has directly related to the sensitivity of tumor tissue. Therefore, predicting the sensitivity of tumors to radiotherapy and chemotherapy plays an important role in the choice of treatment options. The sensitivity of tumor radiotherapy is determined by the level of hypoxia. The DE-MRI study of rectal cancer patients undergoing neoadjuvant chemotherapy showed that the Ktrans value of the treatment response group (judged by tumor staging and tumor regression) before treatment was higher than the nonresponse group chemotherapy. The mechanism and high permeability blood vessels have better oxygenation ability, and chemotherapeutic drugs are easier to enter to play a therapeutic effect.

#### 3.4.4. Application in the Development of Antiangiogenic Drugs

Antitumor angiogenesis-targeted drugs can inhibit the vascular endothelial growth factor receptor (vascular endothelial growth, VEGFR) signal transduction pathway, acting on the angiogenic factors released by endothelial cells or surrounding stromal cells, thereby promoting the normalization of tumor blood vessels. It is a hot spot for targeted tumor therapy in recent years. The quantitative indicators of DE-MRI can accurately assess the inhibition of tumor microvascular permeability and the improvement of tumor vascular normalization by antitumor angiogenesis-targeted drugs. More than 100 items use DE-MRI to evaluate the early clinical stage of antivascular therapy showing that DE-MRI has broad clinical application prospects in evaluating the dynamic changes of tumor blood vessels, exploring the “effective time window” of antiangiogenesis, and monitoring antiangiogenesis efficacy.

## 4. Conclusion

In this paper, dynamic enhanced magnetic resonance imaging technology can be used to effectively explore the diagnosis and clinical application of hematological malignancies. We used Siemens 3.0T to perform MRI and dynamic enhanced MRI on 30 patients with multiple myeloma. The MRI of MM that occurs in the spine is mainly manifested as multiple osteolytic destruction of the spine and extensive osteoporosis. Osteolytic destruction is mainly manifested as trough-like changes or worm-eaten changes, which are diffusely distributed in the vertebral body and appendages. Compared with normal bone marrow, MM's T1WI is mainly low signal, T2WI is high signal, SIRT and T2 fat saturation suppression sequence have fat high signal suppression, and the contrast between the lesion signal and normal bone marrow is more obvious. The enhanced scan is based on its blood supply and different degrees of reinforcement. Most of the selected cases in this group showed this signal's characteristic, and compared with other diseases, the signal characteristic was not specific. The results showed that the diagnostic accuracy of 30 cases of dynamic enhanced MRI was 100%, while the diagnostic accuracy of ordinary MRI was lower than that of dynamic enhanced MRI, p<0.05, and the difference was significant. To sum up, the clinical use of MRI can detect and diagnose MM early, combined with clinical data for comprehensive analysis and diagnosis, which is helpful to formulate effective treatment plans, prolong their survival time, and improve their quality of life. 

The imaging features of the 60 patients with hematological malignancies in this study are mainly as follows: ① The blood density of the patients with hematological malignancies during MRI examination is lower than that of normal patients, but there is no obvious soft tissue damage. ② If the patient's blood vessels are swelling and damaged, the MRI performance is mainly that the edges are relatively clear, and there are many bright areas of different sizes. These bright areas are formed by the destruction of hematological tumor lesions. ③ If there is a soft tissue mass, it will appear on MRI that the signal is generally low, and some are in the state of “salt and pepper sign.” This study showed that the diagnostic sensitivity of MRI in diagnosing hematological malignancies was 65.3%, while the diagnostic accuracy rate was 68.1%, indicating that MRI can still be used as an early detection method for hematological malignancies. However, for some relatively few lesions and special lesions, the diagnosis rate of MRI is not very high. Therefore, dynamic enhanced MRI is needed for another diagnosis, which has higher tissue density and resolution than MRI.

As a noninvasive and dynamic imaging technique for evaluating tumor microcirculation function, the research and clinical application prospects of DE-MRI are very broad. With the development of multicenter research and the cooperation of various interdisciplinary, DE-MRI will be more and more widely used in clinical practice. DE-MRI is one of many MRI techniques for evaluating tumor microcirculation function. Studies have shown that the dynamic parameters of MRI are related to the immunohistochemical markers of tumor angiogenesis and the pathological grade of the tumor. The dynamic parameters after treatment are closely related to the histopathological results and patient survival rate.

## Figures and Tables

**Figure 1:** MRI equipment: (a) principle of magnetic field spin; (b) MRI decay curve; (c) MRI strip.

**Figure 2:** Structure and composition of the 400 MHz MRI spectrometer.

**Figure 3:** Signal recognition of DE-MRI.

**Figure 4:** MRI hematological malignant tumor imaging process.

**Figure 5:** The development process of malignant hematological tumor cells.

**Figure 6:** MRI image of hemangioma. (a, b) DE-MRI showing angiography of hemangioma; (c) nodule changes in lesions; (d) filler angiography of advanced hemangioma.

**Figure 7:** MRI image of liver hemangioma. (a) DE-MRI showing angiography of hemangioma; (b) filling angiography of advanced liver hemangioma.

**Figure 8:** Comparing results of MRI and DE-MRI.

**Figure 9:** Different segments of liver hemangioma MRI.

**Figure 10:** Tumor diagnosis by MRI and DE-MRI.

**Table 1:** Comparison of MRI and DE-MRI.

Common image noise reduction methods	Algorithm advantages	Algorithm disadvantages
MRI	The algorithm is simple, the convolution speed is fast, and it has a good removal effect for Gaussian noise, and so on	Unable to retain complete image information, it is easy to confirm the disease and cause misdiagnosis
DE-MRI	Under the condition that the complete image information is retained to the greatest extent, noise removal is performed to avoid misdiagnosis	The equipment is complex and the running speed is slow

**Table 2:** DE-MRI image features.

Common features	Description	Evaluation
Morphological characteristics	Roundness: the roundness of the lesion Area: the area of the lesion Edge sharpness: average signal gradient at the edge of the lesion Border irregularity: the shape deviation of the edge of the lesion	Important guiding role in the judgment of benign and malignant tumors, and the calculation is relatively simple. Classification effect is not as good as other features.

Texture feature	Contrast: it reflects the sharpness of the image Autocorrelation: it reflects the texture consistency of the image ASM energy: it reflects the uniformity of image grayscale Inverse moment of difference: it reflects the homogeneity of image texture Entropy: it reflects the nonuniformity of image texture	Reflect the texture characteristics of the image. Classifiers trained as features are better than morphological features.

Hemodynamic characteristics	Maximum absorption: the peak of the kinetic curve Peak time: the time required to reach the peak Absorption rate: the absorption rate of the contrast agent Attenuation rate: the rate of attenuation of the contrast agent Enhancement ratio: the ratio of signal strength before enhancement to average signal strength enhancement	The classifier trained as a feature works best.

**Table 3:** Flat sweep.

	T1WI	T2WI	T2-Tirm	DWI (SE-EPI)
TR (ms)	580	4420	8690	3680
TE (ms)	12	96	71	60
FOV (mm)	310	340	420	300
Matrix	310 × 512	330 × 512	360 × 512	128 × 128
Layer thickness (mm)	4	4	4	5
Interval (mm)	1	1	1	2

## Data Availability

The data used to support the findings of this study are available from the corresponding author upon request.
